The article "Phytochemical Constituents, Biological Activities, and Health-Promoting Effects of the Melissa officinalis" was retracted in 2024. Reasons: signs of a paper mill; compromised peer review; unreliable results or conclusions.

# Phytochemical Constituents, Biological Activities, and Health-Promoting Effects of the *Melissa officinalis*

**DOI:** 10.1155/2021/6584693

**Published:** 2021-12-31

**Authors:** Javad Sharifi-Rad, Cristina Quispe, Jesús Herrera-Bravo, Muhammad Akram, Wafa Abbaass, Prabhakar Semwal, Sakshi Painuli, Dmitry Alekseevich Konovalov, Mary Angelia Alfred, Nanjangud Venkatesh Anil Kumar, Muhammad Imran, Muhammad Nadeem, Barbara Sawicka, Piotr Pszczółkowski, Bernadetta Bienia, Piotr Barbaś, Shafi Mahmud, Alessandra Durazzo, Massimo Lucarini, Antonello Santini, Miquel Martorell, Daniela Calina

**Affiliations:** ^1^Facultad de Medicina, Universidad del Azuay, Cuenca, Ecuador; ^2^Facultad de Ciencias de la Salud, Universidad Arturo Prat, Avda. Arturo Prat 2120, Iquique 1110939, Chile; ^3^Departamento de Ciencias Básicas, Facultad de Ciencias, Universidad Santo Tomas, Chile; ^4^Center of Molecular Biology and Pharmacogenetics, Scientific and Technological Bioresource Nucleus, Universidad de La Frontera, Temuco 4811230, Chile; ^5^Department of Eastern Medicine, Government College University Faisalabad, Pakistan; ^6^Department of Life Sciences, Graphic Era (Deemed to be University), Dehradun (248002), Uttarakhand, India; ^7^Uttarakhand State Council for Science and Technology, Vigyan Dham, Dehradun, 248007 Uttarakhand, India; ^8^Himalayan Environmental Studies and Conservation Organization, Prem Nagar, Dehradun, 248001 Uttarakhand, India; ^9^Department of Pharmacognozy and Botany, Pyatigorsk Medical and Pharmaceutical Institute, A Branch of Volgograd State Medical University Ministry of Health of the Russian Federation, Kalinina av.11, Pyatigorsk 357532, Russia; ^10^Department of Chemistry, Manipal Institute of Technology, Manipal Academy of Higher Education, Manipal 576104, India; ^11^University Institute of Diet and Nutritional Sciences, Faculty of Allied Health Sciences, The University of Lahore-Lahore, Pakistan; ^12^Department of Environmental Sciences, COMSATS University Islamabad, Vehari Campus, Pakistan; ^13^Department of Plant Production Technology and Commodities Science, University of Life Sciences in Lublin, Poland, Akademicka 13 Str., 20-950 Lublin, Poland; ^14^The Experimental Station for Variety Assessment of the Central Plant Research Center Uhnin, ZDOO Uhnin, 21-211 Dębowa Kłoda, Poland; ^15^Department of Herbal Medicine, Carpathian State University in Krosno, Poland, Dmochowskiego 12 Str., 38-400 Krosno, Poland; ^16^Department of Potato Agronomy, Plant Breeding and Acclimatization Institute-National Research Institute, Jadwisin Research Center, Poland; ^17^Genetic Engineering and Biotechnology, University of Rajshahi, Rajshahi, Bangladesh; ^18^CREA-Research Centre for Food and Nutrition, Via Ardetina 546, 00178 Rome, Italy; ^19^Department of Pharmacy, University of Napoli Federico II, Via D. Montesano 49, 80131 Napoli, Italy; ^20^Department of Nutrition and Dietetics, Faculty of Pharmacy and Centre for Healthy Living, University of Concepción, Concepción, Chile; ^21^Unidad De Desarrollo Tecnológico (UDT), Universidad De Concepción, Concepción, Chile; ^22^Department of Clinical Pharmacy, University of Medicine and Pharmacy of Craiova, 200349 Craiova, Romania

The article "Phytochemical Constituents, Biological Activities, and Health-Promoting Effects of the Melissa officinalis" was retracted in 2024. Reasons: signs of a paper mill; compromised peer review; unreliable results or conclusions.

## Abstract

Medicinal plants are being used worldwide for centuries for their beneficial properties. Some of the most popular medicinal plants belong to the *Melissa* genus, and different health beneficial effects have already been identified for this genus. Among these species, in particular, the *Melissa officinalis* L. has been reported as having many biological activities, such as antioxidant, antimicrobial, antitumour, antiviral, antiallergic, anti-inflammatory, and also flatulence inhibiting effects. The beneficial properties of the *Melissa officinalis*, also known as “lemon balm herb”, can be related to the bioactive compounds such as terpenoids, alcohols, rosmarinic acid, and phenolic antioxidants which are present in the plant. In this updated review, the botanical, geographical, nutritional, phytochemical, and traditional medical aspects of *M. officinalis* have been considered as well as *in vitro* and *in vivo* and clinically proven therapeutic properties have been reviewed with a special focus on health-promoting effects and possible perspective nutraceutical applications. To evidence the relevance of this plant in the research and completely assess the context, a literature quantitative research analysis has been performed indicating the great interest towards this plant for its beneficial properties.

## 1. Introduction

Medicinal plants and herbs have been used worldwide in the management of different diseases [1, 2]. The search for new antibacterial, antiviral, anticancer agents from natural sources has been intensified due to the reduction of currently available therapy in subjects who do not qualify for conventional pharmacological therapy and the emergence of drug-resistant strains [3, 4]. Recently, the nutraceutical area has been exploited playing a key role in the development of new phytocomplex derived from food and plant-derived compounds [5, 6].

An example of popular medicinal plants with recognized beneficial effects on human health belongs to the *Melissa* genus [7]. Botanically, this plant can be identified as follows: genus *Melissa* L. belongs to kingdom: Plantae, family: Lamiaceae, and subfamily: Nepetoideae, with numerous species, four of which are *Melissa axillaris* (Benth.) Bakh. f., *Melissa flava* Benth., *Melissa officinalis* L. (lemon balm), and *Melissa yunnanensis* C.Y. Wu & Y.C. Huang which is recognized worldwide for its relevance [8, 9]. These species are found in the area from Central Asia, Western Asia, Southern Europe, and Northern Africa up to the islands of Macaronesia [8]. Only one species grows in Europe—the M*. officinalis* known as lemon balm. In nature, these plants grow in bright thickets [10].

The article "Phytochemical Constituents, Biological Activities, and Health-Promoting Effects of the Melissa officinalis" was retracted in 2024. Reasons: signs of a paper mill; compromised peer review; unreliable results or conclusions.

Currently, this most popular and known species, the *M. officinalis*, is cultivated around the world [11–13]. Even if the *M. officinalis* is indigenous to Southern Europe, the Mediterranean region, Western Asia, and North Africa, this species is now cultivated worldwide. In India, lemon balm is cultivated in Kashmir, Uttrakhand, and some parts of South India. There are two subspecies: *M. officinalis* subspecies *M. officinalis*, the commonly cultivated lemon balm; and *M. officinalis* subspecies *altissima*, naturalized in New Zealand and known as the bush balm. The *M. officinalis* subspecies *officinalis* is known for its lemon fragrance [12, 14].

Nowadays, the increasing demand for medicinal plants and herbs triggers the interest in quality and safety aspects since herb and plants pathogens, e.g., microfungi, could cause serious health issues if present in these plants decreasing also their quality [15, 16]. Species like *Fusarium* sp., *Alternaria* sp., and *Penicillium* sp. can produce secondary metabolites (mycotoxins) which may represent a healthy treat as it happens also in plants, food, and feed contaminated by these metabolites which represent a challenge for the decontamination due to their presence and their identification (Nazhand et al., 2020; Santini et al. 2009; Mikusova et al. 2013; Mikusova et al. 2010; Santini et al., 2009).

## 2. *Melissa officinalis* and Its Health Benefits: Literature Quantitative Research Analysis

A search for *Melissa officinalis* and its relationship with health was carried out employing the Scopus database. The Scopus online database (https://www.scopus.com/home.uri, accessed on 4 September 2021) was utilized to extract bibliometric data using the search string: TITLE-ABS-KEY (“*Melissa officinalis*” OR “lemon balm” AND “Health∗”).

Publications mentioning the relevant words or their derivatives in the title, abstract, or keywords were identified throughout the applied search strategy [17]. The parameters evaluated were as follows: trends of publications, document type, authorship, and country/region. For the basic analyses, the functions of the Scopus web online platform named “Analyze” and as “Create Citation Report” were utilized. Moreover, the “full records and cited references” were exported to VOSviewer software for additional processing [18].

The article "Phytochemical Constituents, Biological Activities, and Health-Promoting Effects of the Melissa officinalis" was retracted in 2024. Reasons: signs of a paper mill; compromised peer review; unreliable results or conclusions.

The terms/words utilized in the titles, abstracts of publications, and keywords of publications were analyzed by the VOSviewer software (v.1.6.16, 2020); the paragraphs were broken down into words and phrases and linked to the publications' citation data, to visualize the results as bubble map. In this term map, the bubble size indicates how frequently a term is mentioned in the articles. Two bubbles are positioned more closely to each other reflecting that the terms coappeared more often in the selected publications. The average citations per publication (CPP) is given by the colour of a bubble. To simplify the bubble map, words/terms that appeared in at least 5 of the publications were analyzed and visualized. Of the 5772 keywords, 436 met the selected threshold, and 3 of them were manually excluded.

Two hundred seventy publications were returned by the search: they covered the time range from 1984 to 2021 and were cited collectively by 5682 documents. Publications trends of the *Melissa officinalis* and health research are reported in Figure 1.

The distribution of the types of documents relative to the publications retrieved is shown in Figure 2. “Article” accounts for 75.9% and “Review” for 18.1%, followed by Book Chapter” (1.9%) and “Conference Paper” (1.5%). The most cited “Article” is a placebo-controlled trial for studying the value of aromatherapy with essential oil of *Melissa officinalis* for agitation in people with severe dementia, whereas the most cited “Review” is addressed on Alzheimer's disease and vascular dementia in developing countries, with regard on the use of traditional diet and medicinal plants.

Figure 3 reports the most productive authors.

Figure 4 reports, respectively, the most productive countries/territories. Regarding countries/territories, the United States (*n* = 30) was the most productive country, followed by Iran (*n* = 28) and the United Kingdom (*n* = 27).

Four hundred and the thirty-third of terms in total were obtained from the literature quantitative analysis on publications, and they are visualized as a term map shown in Figure 5. Plant extracts, *M. officinalis* extract, medicinal plants, phytotherapy, herbal medicine, and traditional medicine are among the top recurring terms.

## 3. Traditional Medicinal Uses

*M. officinalis* is a medicinal plant that has been used for a long time in different ethnomedical approaches especially in traditional medicine for the treatment of several diseases. The traditional uses of *M. officinalis* have been reported mostly in European Countries, the Mediterranean region, and the Middle East Countries.

The article "Phytochemical Constituents, Biological Activities, and Health-Promoting Effects of the Melissa officinalis" was retracted in 2024. Reasons: signs of a paper mill; compromised peer review; unreliable results or conclusions.

Records concerning the use of *M. officinalis* date back over 2000 years, with entries in the Historia Plantarum (approximately 300 B.C.). Its use has been exploited for the treatment of many health syndromes including neurological, central nervous system, cardiovascular, antimicrobial, antimalignant, antidepressant, and respiratory and also as a memory enhancer for dementia-affected subjects. In the seventh century, its cultivation and use spread throughout Europe [19]. An early recommendation by Paracelsus (1493–1541) suggested that it could be used for “all complaints supposed to proceed from a disordered state of the nervous system” [20].

*M. officinalis* is reputed to alleviate melancholia and neuroses, and the plant was considered to promote long life and to restore memory in traditional European medicine [21]. In 1679, Lonicerus claimed that *M. officinalis* (the aerial parts) taken on an empty stomach quickens the senses, brightens the mind, and improves the memory. It aids shaking limbs caused by stroke and helps retrieve the lost ability to speak [22, 23]. Moreover, in 1751, the herbalist John Hill described *M. officinalis* as “good for disorders of the head and stomach” [21], and in the Ayurveda holistic medicine approach, it was claimed that *M. officinalis* sharpens memory [24]. *M. officinalis* is a cultivated and introduced herb in the Callejon de Huaylas (Peru), used as a sedative, and hypotensive [25]. Herbal medicine has been traditionally practiced by indigenous healers in Bolivia for hundreds of years, an area where due to the great geographical and ecological diversity, thousands of native plants are utilized against different types of diseases [26].

Often the traditional use of *M. officinalis* is mostly combined with other medicinal plants. For instance, around 400 prescriptions are containing *M. officinalis* in Iranian Traditional Medicine [27]. An ethnobotanical study of the medicinal use of wild and cultivated plants in the middle, southern, and western Bosnia and Herzegovina showed that *M. officinalis* is part of the combined teas for the increase of digestion (with *Acorus*, *Foeniculum*, *Matricaria*, and *Mentha*), a decrease of spasms (with *Agrimonia*, *Frangula*, *Mentha*, *Teucrium chamaedrys*, and *Teucrium montanum*), and insomnia (with *Robinia*) [28].

Medicinal plants which can be used as tools against anxiety and as antidepressant drugs according to the ethnobotanical knowledge in Shahrekord (Iran) include *M. officinalis*, proven to be effective on anxiety and depression [29]. In the Unani system of medicine, its grass and seeds are used in epilepsy, paralysis, Bell's palsy, arthritis, mastitis, and halitosis; its syrup and distillate are made for different ailments [30].

The article "Phytochemical Constituents, Biological Activities, and Health-Promoting Effects of the Melissa officinalis" was retracted in 2024. Reasons: signs of a paper mill; compromised peer review; unreliable results or conclusions.

*M. officinalis* is used as a sedative, and for its digestive properties in Serbia, it is used for nervous anxiety, depression, tension headaches, and indigestion (as a tea-like beverage that is drunk after a meal). It is also used for diseases related to the liver and gallbladder, jaundice, and complaints related to the heart and blood vessels, and it is administered as an infusion (tea). As an example of its use, a recipe of a tea blend for strengthening nerves consists of equal quantities of lemon balm, valerian, hops, hawthorn, wild thyme, and peppermint. For peaceful sleep, pillows are filled with the dried aerial parts (northern and western Serbia). It is also used to lure bees—beekeepers rub hives (in eastern Serbia) [31].

An ethnobotanical survey of the wild plants of Lebanon showed that *M. officinalis* is harvested and used as a spice, herbal tea, condiment, medicinal plant, and in perfumes [32]. In Central Italy, *M. officinalis* shoots are used in alcoholic beverages [33]. Ethnobotanical evidence suggests that the herb of *M. officinalis* is used for the skin and body care. Lemon balm hydrosol is added to clay masks for skin healing. Fresh leaves add a nice flavour to many dishes, oils, vinegar, and herbal liqueurs. Fresh or dried leaves are used to prepare a refreshing tea, consumed either cold or hot. The fresh leaves and flowers are used for the stuffing of vegetables, fruit salads, bean dishes, meat, and fish [12]. It is noteworthy that the traditional use of this plant is similar in different cultures: for example, treatment of mental disorders, especially anxiety and depression, memory improvement, and relief of heart disease. As can be seen from the data reported in Table 1, the above-ground part and the leaves of the plant have traditionally been used more often; from them, mainly, an infusion, tea, or decoction can be prepared.

Table 1 summarizes some relevant information on the traditional use of *M. officinalis* in different countries.

## 4. Chemical Composition

The most important class of plant components are alkaloids, tannins, flavonoids, saponins, and phenolic compounds [10, 12, 79]. The variety of these bioactive molecules makes them a promising candidate for the development of nutraceuticals and cosmeceuticals [10, 80]. This plant and its parts can be used in the food, pharmaceutical, cosmetic, and other industries which are interested in aromatic plants and essential oils.

### 4.1. Polyphenols

Regarding the polyphenolic profile of extracts, Awad et al. [81] isolated rosmarinic acid, ursolic acid, and oleanolic acid from the methanol extract of aerial parts of *M. officinalis*.

The article "Phytochemical Constituents, Biological Activities, and Health-Promoting Effects of the Melissa officinalis" was retracted in 2024. Reasons: signs of a paper mill; compromised peer review; unreliable results or conclusions.

Astani et al. [82] isolated caffeic acid, *p*-coumaric acid, and rosmarinic acid. Nitric acids A and B, antioxidant active compounds, have been identified in the dried leaf of *M. officinalis* by Kamdem et al. [83] and quantified. The leaves were extracted in 70% ethanol, which resulted in the following compounds quantified using liquid chromatography-mass spectrometry (LC-MS): gallic acid, chlorogenic acid, caffeic acid, rosmarinic acid, ellagic acid, rutin, isoquercitrin, quercetin, and kaempferol. Aubert et al. [84] identified the following compounds from hydroethanolic leaf extract of *M. officinalis* using LC-MS: tartaric acid, quinic acid, malic acid, citric acid, succinic acid, danshensu, caftaric acid, salicylic acid, caffeic acid, lithospermic acid A, chicoric acid, luteolin 3′-*O*-*β*-D-glucuronide, rosmarinic acid, 3′-*O*-(8′-*Z*-caffeoyl)rosmarinic acid, and ethyl caffeate.

Another example has been reported by Binello et al. [85] where an efficient and selective green extraction of polyphenols from lemon balm has been proposed using ultrasound and microwave-assisted extraction protocols. Their efficiency and selectivity have been compared: rosmarinic acid was the main component of the phenolic fractions in all cases, whereas ethanol was the best solvent for both ultrasound and microwave-assisted extraction procedures [85].

### 4.2. Essential Oil

Concerning the characterization of the essential oil, several works studied the composition of the aerial flowering parts of *M. officinalis* [80, 86–88].

For instance, Acevedo et al. [80] isolated the following essential oils: eugenol, caryophyllene, *α*-caryophyllene, 3-methyl-4-isopropyl phenol, and germacrene D. Abdellatif et al. [89, 90] hydro distilled the dried leaves of *M. officinalis* and identified the following essential oils using gas chromatography coupled to mass spectrometry (GC-MS): 1-octen-3-ol, 6-methyl-5-hepten-2-one, myrcene, (*Z*)- and (*E*)-*β*-ocimene, linalool, *n*-nonanal, *cis*- and *trans*-rose oxide, *trans*-limonene oxide, camphor, citronellal, *cis*-chresontynol, menthol, isomenthol, nerol, neral, piperitone, geraniol, geranial, dihydrocitronellol acetate, *α*- and *β*-cubebene, geranyl acetate, *α*-copaene, *β*-caryophyllene, *α*-humulene, germacrene D, (*E*)-*β*-ionone, valencene, (*E*)-nerolidol, caryophyllene oxide, 1-hexadecene, 14-hydroxy-9-epi-(*E*) caryophyllene, *n*-eicosane, *n*-heneicosane, methyl citronellate, and camphene. Barakat et al. [91] identified the following compounds by hydrodistillation of dried leaves of *M. officinalis* using GC-MS: (*E*)-ocimene, *α*-campholenal, pinocarvone, terpinen-4-ol, cumin aldehyde, thymol, *p*-mentha-1,4-diene-7-ol, *α*-copaene, *β*-bourbonene, panasinsene, (*E*)-caryophellene, amorpha-4,11-diene, *γ*-muurolene, elemol, caryophellene oxide, humulene epoxide II, elemol acetate, *α*-terpinolene, trans-pinocarveol, *cis*-chrysanthenol, (*E*)-citral, carvacrol, decadienal, *α*-copaene, *β*-bourbonene, and isotorquatone. Efremov et al. [92] extracted the essential oils by exhaustive water and steam distillation from the above-ground part of *M. officinalis*.

The article "Phytochemical Constituents, Biological Activities, and Health-Promoting Effects of the Melissa officinalis" was retracted in 2024. Reasons: signs of a paper mill; compromised peer review; unreliable results or conclusions.

Rehman et al. [93] identified from *M. Officinalis* fresh leaves using the headspace solid-phase microextraction (HS-SPME) coupled with GC-MS with the following compounds, all with interesting activity: *β*-pinene, artemiseole, 1-octen-3-ol, 3-octanol, 6-methyl-5-hepten-2-one, D-3-carene, (*Z*)-*β*-ocimene, linalool, *cis*-rose oxide, *trans*-rose oxide, *cis*-verbenol, limonene oxide, citronellal, isopulegone, myrtenol, citronellol, geraniol, (*Z*)-citral, methyl geranate, (*E*)-citral, citronellyl acetate, *α*-copaene, geranyl acetate, *β*-caryophyllene, *α*-bergamotene, *α*-humulene, germacrene D, *α*-farnesene, and D-cadinene. In the perspective of an eco-friendly sustainable procedure, it is worth to mention the work of Khalili et al. [94], which reported the solvent-free extraction of essential oils from *M. officinalis*. The compounds identified by GC-MS are linalool, (*Z)*- and (*E*)-citral, neryl acetate, *β*-bourbonene, *β*-bourbonene, *α*-humulene, germacrene D, *α*-muurolene, and caryophyllene oxide.

## 5. Biological Activities of *Melissa officinalis: M*olecular Evidences from Preclinical Studies

The biological properties of the lemon balm herb can be associated with the presence and combined action of bioactive compounds such as terpenoids, rosmarinic acid and phenolic antioxidants. The most important bioactive compounds from *M officinalis* and their correlation with biological activities are shown in Figure 6.

### 5.1. Effects on the Central Nervous System

#### 5.1.1. Neuroprotective

In several *in vivo* and *in vitro* studies, the neuroprotection and beneficial treatment of several nervous disorders were attributed to the administration of *M. officinalis*.

Methanolic extract of *M. officinalis* administered to PC12 was reported to provide cell protection against H_2_O_2_ toxicity in lactate dehydrogenase (LDH) and 3-(4,5-dimethylthiazol-2-yl)-2,5-diphenyltetrazolium bromide) (MTT) assay [95]. Moreover, reduction in the intracellular formation of reactive oxygen species and neuroprotection was attributed to the administration of aqueous and methanol extracts *M. officinalis* [96]. Lemon balm was reported to have neuroprotective activity against 3,4-methylenedioxymethamphetamine-induced cell apoptosis in response to free radicals.

The article "Phytochemical Constituents, Biological Activities, and Health-Promoting Effects of the Melissa officinalis" was retracted in 2024. Reasons: signs of a paper mill; compromised peer review; unreliable results or conclusions.

Soodi et al. [97] carried out an *in vivo* study on rats to validate the significant effect of *M. officinalis* as a potential agent for improving brain health. The study determined that the 80% ethanol extract of *M. officinalis* improved memory in induced memory-impaired clinical rats and concluded that *M. officinalis* extract has probable therapeutic potential in alleviating memory loss.

#### 5.1.2. Antidepressant

Ethanolic extract of *M. officinalis* was orally administered in three different concentrations of 30, 100, and 300 mg/kg on a period of 10 days to Wistar rats and forced swimming and elevated plus-maze, and open field tests evaluated their behavioural effects [98]. Moreover, comparative effects against diazepam and fluoxetine were also evaluated. In the elevated plus-maze test, the percentage results in rats with subacute *M. officinalis* ethanol extract were remarkably higher than that in vehicle-treated animals but similar as in the diazepam-treated group, irrespective of the treatment duration. In the forced swimming test, the duration of immobility was reported lower in rats treated with the *M. officinalis* than that of the vehicle-treated group. In the 10-day treatment period, the antidepressant activity of fluoxetine was significantly higher than that of lemon balm [98].

#### 5.1.3. Anxiolytic

Anxiety is a pathological emotional state characterized by anxiety, fear of the possibility of imminent danger or failure and over time natural remedies have proven beneficial [4, 99, 100]. Studies have shown that the anxiolytic effect of *M. officinalis* is dose dependent, and the responsible biocompounds are rosmarinic acid, pentacyclic triterpenes, and oleanolic and ursolic acids. Methanolic extract of *M. officinalis* was administered to the rat brain [101]. Rosmarinic acid, among the main components of the *M. officinalis*, was reported to have extensive *γ*-Aminobutyric Acid Transaminase (GABAT) inhibition medicinal properties. *In vivo* administration of aqueous extract of *M. officinalis* along with *P. caerulea* was reported to demonstrate anxiolytic activity through reduction in corticosterone (physiological stress mediator) level [27, 102, 103].

### 5.2. Antidiabetic

Chemical constituents of *M. officinalis*, oleanolic acid were reported to have potential antidiabetic pharmacological activity by survival and preservation of pancreatic *β*-cells along with protection against diabetic complications. Hence, lipophilic triterpenoids in combination with the ethanolic extract of the plant have been proven as latent antidiabetic agents [27, 102].

The article "Phytochemical Constituents, Biological Activities, and Health-Promoting Effects of the Melissa officinalis" was retracted in 2024. Reasons: signs of a paper mill; compromised peer review; unreliable results or conclusions.

Ethanolic extract of *M. officinalis* (0.6 mg/mL) was reported to induce cell-specific peroxisome proliferator-activated receptor (PPAR) gene expression to human primary adipocytes. However, replication of the same effect in clinical conditions needs further studies with lower doses which are more likely to be administered in humans [104]. Ethanolic extract of *M. officinalis* ethanol (200 mg/kg) was administered to obese mice with known case of insulin resistance for 6 weeks, and a significant reduction in glucose level, weight reduction, and insulin resistance was reported [105].

Alcoholic extract of *M. officinalis* has been reported to have antihyperlipidemic effects through inhibition of cholesterol synthesis and its secretion [106]. Moreover, the ethanolic leaf extract of *M. officinalis* was reported to treat insulin resistance, plasma triglyceride, hyperglycemia, and dyslipidemia in rats through activation of peroxisome proliferator-activated receptors which in turn regulates lipid and glucose metabolism in the body. Hence, ethanolic extract of lemon balm was reported to have potential activity in the prevention and treatment of diabetes mellitus (type-2) and hyperlipidemia [107, 108].

Recently, Lee et al. [109] indicated that a herbal extract of *M. officinalis* not only inhibits visceral obesity but also attenuates the increased fasting blood glucose, impaired glucose tolerance, and pancreatic dysfunction in female obese mice.

### 5.3. Cardioprotective

*M. officinalis* was reported to have significant cardiovascular effects in heart palpitations along with significant cardioprotective and cardiac tonic activities. This effect is due to the presence of saponins and alkaloids. The cardioprotective effects of aqueous extracts of leaves of *M. officinalis* along with *Lippia alba* (Mill.) (http://N.E.Br). ex Britton & P.Wilson and *Cymbopogon citratus* (D.C.) Stapf (concentrations, 0.038, 0.38, 3.8 and 38 mg) was reported in an *in vivo* study on 21 male adult rats to evaluate their activity upon heart rate and cardiac contractile force. The statistical evaluation showed a significant reduction in cardiac rate through muscarinic receptor stimulation while no effect was reported to alter cardia contractility force [110].

Pharmacological evaluation *M. officinalis* was mainly focused on its antiarrhythmic activity. The administration of ethanolic extract of lemon balm was reported to reduce ventricular fibrillation, tachycardia, and premature beats in CaCl_2_-induced arrhythmias [111]. *β*-Adrenergic antagonistic activity of lemon balm was reported to have antidysrhythmic activity and induce bradycardia [27, 102].

The article "Phytochemical Constituents, Biological Activities, and Health-Promoting Effects of the Melissa officinalis" was retracted in 2024. Reasons: signs of a paper mill; compromised peer review; unreliable results or conclusions.

### 5.4. Anti-Inflammatory

Reduction in inflammation-induced edema in rat paws has been attributed to the administration of aqueous extract of lemon balm. In addition, the administration of ethanolic extract of *M. officinalis*, mainly attributed to rosmarinic acid content, was reported to exert antinociceptive effects by inhibiting the L-arginine-nitric oxide pathway and activating the cholinergic system [27]. *M. officinalis* ethanol extracted powder mixed with corn starch in 1000 mg capsule form was administered to test the group having dysmenorrheal [112]. The severity of pain was significantly reduced from 7.63 to 2.00 in the second menstrual cycle. A remarkable result difference in the first and second menstrual cycle was reported respective to the severity of the pain [113].

### 5.5. Anticancer

A comparative study of five different extracts of *M. officinalis* was conducted to explore the anticancer effects of this medicinal plant on cell lines by Magalhães et al. [114]. The outcomes of this study sign posted that tumour cells growth was inhibited by employing five different extracts on three types of human tumour cell lines depending on the concentration of *M. officinalis* in the extract. The highlights of this study also revealed an inhibitory effect on tumour cell growth by ethanolic extract due to the presence of rosmaricinic acid, with potent penetration power and endorsed *M. officinalis* as a source of bioactive composites with antitumour potential.

Another study was conducted on human colon carcinoma cells to sensitize the *M. officinalis* as a dietary intervention and as a pharmaceutical plant by [115]. The study evidenced that lemon balm methanolic extract prevents the propagation of colon carcinoma cells and self-induce apoptosis in HT-29 and T84 human colon carcinoma cell lines after 3 to 4 days. Another study investigated lemon balm as an antiproliferative agent on different types of cell lines of breast cancer. The outcomes showed that *M. officinalis* extracts have anticancer potential against breast tumours in the cell culture line, due to the presence of the phenolic acids [115]. The recent work of Ghiulai et al. [116] reported how lemon balm extracts prevent breast cancer progression *in vitro* and i*n vivo* using the chorioallantoic membrane assay.

### 5.6. Antimicrobial

The discovery and introduction of antibiotics in medicine had a beneficial effect on the control of infectious diseases [117, 118]. Unfortunately, excessive use of antibiotics has been accompanied by the rapid emergence of resistant bacterial strains that are difficult to eradicate and undesirable side effects [7, 119]. As a result, the researchers focused on the discovery of natural bioactives with antibacterial effect but with fewer side effects [120]. Leaf extract of *M. officinalis* was reported to have antimicrobial activity against bacterial strains of 13 test microbes. The antibacterial effect of the essential oil of M. officinalis was due to the content of aldehydes, ketones, and monoterpenes [121, 122]. Gram-positive bacteria were reported to exhibit more sensitivity to plant extract than Gram-negative bacteria.

The article "Phytochemical Constituents, Biological Activities, and Health-Promoting Effects of the Melissa officinalis" was retracted in 2024. Reasons: signs of a paper mill; compromised peer review; unreliable results or conclusions.

### 5.7. Antiviral

Oral herpes is caused by the herpes simplex virus type 1 (HSV-1), which enters the body and reactivates, causing an unsightly lesion on the surface of the lips, during periods when the immune system is weakened [15, 123].

A special biological action of *M. officinalis* is antiviral on the herpes virus herpes simplex 1 (HSV-1). This antiviral activity is determined by polyphenolic acids and their derivatives, compounds present in the aqueous extract obtained from the *M. officinalis* leaves. The mechanism of antiviral action involves interaction between polyphenolic compounds, viral proteins, and cell membrane proteins. There is a blockage of membrane receptors (from the cells of the mucosa where the rash is to occur) by polyphenolic compounds, thus preventing the adhesion of the herpes virus-1 to the cell wall and, thus, the beginning of the viral infection spread cycle, after transduction [124].

### 5.8. Antithyroid Activity

The thyroid gland produces thyroid hormones, which have many functions in the body, one of which is to regulate metabolism [125]. Thyroid diseases are treated with medication and surgery, but there are also natural remedies that can be used for treating these [126]. In vitro experiments showed an antithyroid activity for aqueous extracts of *M. officinalis* leaves. Thus, the conversion of T4 to T3, depending on the dose, was observed by action on iodothyronine deiodinase obtained from rat liver microsomes [127]. The effects are dose dependent and are due to caffeic, rosemary, and chlorogenic acids. Compared to some conventional antiviral drugs (idoxuridine), these bioactive compounds from *M. officinalis* cause a shortening of the healing period of herpes lesions and a decrease in the recurrence of viral infection. [127].

## 6. Clinical Studies

Recently, a research group from Iran reported the effects of *M. officinalis* leaves (in the form of *Melissa* capsule) on anxiety and sleep quality in patients undergoing coronary artery bypass surgery. The clinical trial was conducted on 80 patients, and all patients were given herbal drugs (500 mg of *M. officinalis* leaves) while the placebo control group was given 500 mg of wheat starch three times a day. The results of seven days of treatment with *M. officinalis* reduced the level of anxiety (49%) and improved the sleep quality (54%) in patients after coronary artery bypass surgery [128].

The article "Phytochemical Constituents, Biological Activities, and Health-Promoting Effects of the Melissa officinalis" was retracted in 2024. Reasons: signs of a paper mill; compromised peer review; unreliable results or conclusions.

Watson et al. [129] from Sydney reported the effects of *M. officinalis* essential oil in the treatment of agitated behaviour in older people with and without dementia. A total of 39 nursing home residents with dementia and 10 without dementia participated in this study. Participants were treated with essential oil for two weeks followed by a two-week washout period before commencing the subsequent treatment. Essential oil of *M. officinalis* exhibited more effective in reducing agitation in people without dementia (Trial registration no: ACTRN12614000130662) [129].

Tavares-Silva et al. [130] from Brazil demonstrated the efficacy of *M. officinalis* and *Phytolacca decandra* L. and its combination in the treatment of possible sleep bruxism in children. The clinical trial was conducted on 52 children, based on the parent's report of sleep bruxism. The results of 30 days of treatment with *M. officinalis* reduced the possible sleep bruxism in children, while its combination with *P. decandra* did not improve the results (Trial registration any: NCT02870543) [130].

Nayebi et al. [131] reported the impact of *M. officinalis*-based products in diabetic patients (affected by Type 2 diabetes). The clinical trial was conducted on 37 dyslipidemic diabetic patients, and all the patients were treated with *M. officinalis* or placebo at the dose of two 500 mg, administered as capsules daily in a 3-month timeframe. *M. officinalis* significantly decreased the serum level of triglyceride, and no other metabolic changes were recorded when compared with the control group (Trial registration no: IRCT2015112625251N1) [131].

Asadi et al. [132] demonstrated the antidiabetic activity of hydroalcoholic extract of *M. officinalis* in type 2 diabetic patients. The clinical trial was performed on 62 patients receiving the dose of Melissa officinalis or placebo (700 mg per day) twice for 12 weeks. The results of this study indicated that *M. officinalis* extract causes a significant change in fasting blood sugar level, glycated haemoglobin (HbA1c), and systolic blood pressure in comparison with the placebo group. The herbal capsule of *M. officinalis* was safe and effective in enhancement of lipid profile, glycemic control, and reduction of inflammation (Trial registration number: IRCT201701162709N41) [132].

Darvish-Mofrad-Kashani et al. described the efficacy and safety of *M. officinalis* in the improvement of hypoactive sexual desire disorder in women [133]. A total of 89 women suffering from the disease participated in the study and were treated with the aqueous extract of *M. officinalis* or placebo with a dose of two 500 mg capsules per day for 4 weeks. The results of the 4-week study demonstrated that *M. officinalis* extract significantly increased the scores of desire, arousal, lubrication, orgasm, satisfaction, and pain compared to placebo in hypoactive sexual desire disorder in women [133]. Another research group from Iran also discovered the combination of *M. officinalis* and *Nepeta menthoides* Boiss. & Buhse in sleep disorder [134]. A total of 102 patients participated in this study, but only 80 were selected after the screening. Selected patients have been treated with the dose of 1000 mg of *M. officinalis* plus 400 mg of *N. menthoides* or a placebo for four weeks. The 4-week trial demonstrated that a combination of both showed significant activity against insomnia (Trial registration number: IRCT2015040621592N2) [134].

The article "Phytochemical Constituents, Biological Activities, and Health-Promoting Effects of the Melissa officinalis" was retracted in 2024. Reasons: signs of a paper mill; compromised peer review; unreliable results or conclusions.

Oral administration of *M. officinalis* and its impact on biomarkers of oxidative stress, inflammation, and lipid profile in chronic stable angina patients were reported by Javid et al. [135]. The clinical trial was conducted in 80 patients with chronic stable angina and treated with a dose of 3 g per day for 8 weeks. The oral administration of *M. officinalis* powder significantly improved the lipid profile, malondialdehyde (MDA), high sensitivity c reactive protein (hs-CRP), and PNO1 in chronic stable angina patients (Trial registration number: IRCT2016052928152N1) [135]. Perry et al. [136] from the UK reported the effects of a combination of *Salvia officinalis* L., *Rosmarinus officinalis* L., and *M. officinalis* (SRM) against enhancement of memory and brain function in a healthy person. The results of the study demonstrated that an oral administration of SRM combination at the dose of 5 mL two times per day for 2 weeks is more effective when compared with a placebo [136]. Martinelli et al. [137] from Italy reported the effectiveness of *Matricaria chamomilla* L., *M. officinalis* and tyndallized *Lactobacillus acidophilus* (HA122) in infant colic. A total of 176 patients completed the 28-day trial, and crying time was significantly lower in groups A (who was given *M. chamomilla*, *M. officinalis*, and tyndallized *L. acidophilus*) and B (who was given *Lactobacillus reuteri*) when compared with group C (who was given simethicone) at the 28th day. The administration of *M. chamomilla*, *M. officinalis*, and tyndallized *L. acidophilus* showed more effectiveness than that of simethicone in infant colic (Trial registration number: NCT02708238) [137]. Other important clinical trials of *Melissa* genus have been summarized in Table 2.

The article "Phytochemical Constituents, Biological Activities, and Health-Promoting Effects of the Melissa officinalis" was retracted in 2024. Reasons: signs of a paper mill; compromised peer review; unreliable results or conclusions.

## 7. Safety Data

The safety aspects of *M. officinalis* were testified by Haybar et al. [147]. Furthermore, verdicts of potential open-label research trials did not impart any adverse effects after oral consumption of M*. officinalis* 600 mg per day dose. The anxiolytic effects of *M. officinalis* do not affect the circadian activity and are not accompanied by benzodiazepine-specific reactions. However, doses higher than 600 mg extract/day can increase anxiety and negatively affect mood [140].

The outcomes of two more further clinical studies showed no antagonistic effects among the different treatments of experimental studies [146]. Opposing the aforementioned outcomes of different researchers, some other clinical trials observed adverse effects of *M. officinalis* consumption.

A controlled randomized study described cases of vomiting, faintness, wheezing, hyper activeness, abdominal cramps, and queasiness after drinking 60 drops of *M. officinalis* extract in a 60 days trial [113]. Alijaniha et al. [111] also reported a significant increase in hunger after the *M. officinalis* administering. The 1200 mg dose of *M. officinalis* resulted in causing headache, skin irritation, burning sensation, increased palpitation rate, and hormone inhibition, particularly thyroid hormone as reported by Ulbricht et al. [148]. In conclusion, utmost attention should be given in case of long-term utilization of this herbal plant concerning the therapy of the above-cited health associated conditions.

## 8. Therapeutic Perspectives

“Nutraceutical Science” represents a great challenge for the future [149, 150]. An emerging direction was given by nanonutraceuticals that assure their value at a nanolevel as well as safety and efficacy [151, 152]. Nowadays, some emerging applications of nanotechnologies to *Melissa* extracts have been reported [153–155]. For instance, Rostami and Esfahan [155] described the development of a smart edible nanocomposite based on mucilage of *M. officinalis* seed/montmorillonite/curcumin. This may open a novel frontier for the use of this plant and understanding the mechanism of action of its components.

Therapeutic limitations of bioactive natural compounds are represented by possible interactions with other drugs [2, 156]. Regarding drug interactions, *M. officinalis* may have a sedative effect if combined with alcohol, over-the-counter sleep treatments, or prescription sedatives such as clonazepam, lorazepam, phenobarbital, and zolpidem. It may also interact with other medicines levothyroxine (to treat thyroid disorders), warfarin, clopidogrel (anticoagulants), travoprost (antiglaucoma), tamoxifen, and irinotecan (cytostatics). [157].

The article "Phytochemical Constituents, Biological Activities, and Health-Promoting Effects of the Melissa officinalis" was retracted in 2024. Reasons: signs of a paper mill; compromised peer review; unreliable results or conclusions.

## 9. Concluding Remarks

Considering the naturally occurring bioactive molecules with a beneficial potential that can be obtained from plants and herbs, the *Melissa officinalis* is one of the widely used medicinal herbs worldwide. Based on scientific data, *M. officinalis* can be used traditionally for the treatment of several diseases with less toxicity and side effects to support or, in the same cases, as an adjuvant to the conventional pharmacological therapy. The recent researches supported the use of *M. officinalis* for the treatment of certain diseases. Based on this, more researches should be carried out to explore the therapeutic and nutraceutical potential properties of *M. officinalis*. Nevertheless, there is a need for further *in vivo* and *in vitro* research and clinical trials to better understand the related mechanisms of action in the treatment of various diseases.

## Figures and Tables

**Figure 1:** Publication and citations trends of *Melissa officinalis* and health research (bibliometric data were extracted from the Scopus online database).

**Figure 2:** Distribution of type document (bibliometric data were extracted from the Scopus online database).

**Figure 3:** Most productive authors (bibliometric data were extracted from the Scopus online database).

**Figure 4:** Most productive countries/territories (based on data from Scopus).

**Figure 5:** Term map for relationships of *Melissa officinalis* and health research. The number of publications was represented by bubble size. The citations per publication (CPP) was given by bubble colour. Two bubbles are closer to each other reflecting that the terms coappeared more frequently (bibliometric data were extracted from the Scopus online database and elaborated by VOSviewer software).

**Figure 6:** Summarized scheme with the most important bioactive compounds from *M officinalis* and their correlation with biological activities.

**Table 1:** Traditional uses of *Melissa officinalis* in different Countries.

Country/region	Organ/part of plant	Mode of application	Traditional uses	References
Argentina/San Martin de los Andes	—	—	Sedative	[34]
Austria	Leaves	Internal as tea, external essential oil	Treatment of diseases of the gastrointestinal tract, nervous system, liver and bile; food	[35]
Bolivia/Qampaya	Leaves	Infusion	Psychological problems, heart problems	[26]
Bosnia and Herzegovina/Javor Mountain	Aerial parts	Infusion	Insomnia, digestive disorders; spasms, respiratory infections	[36]
Brazil/Santa Catarina	Leaves	—	Colic pain in babies, gastrointestinal, to reduce blood pressure, influenza	[37]
Brazil	Leaves	Decoction	Calmative, migraine, sedative	[38]
Bulgaria	Leaves	Decoction	Sedative, tranquillizer	[39]
	Herb	Decoction	Hypertonia	
	Herb	Decoction	Improves appetite	
Catalonia/L'Alt Emporda and Les Guilleries	Leaves	Infusion	Sedative	[40]
Denmark	Aerial parts	—	Against sleeplessness caused by heartbreak; against melancholy and sadness	[27, 41]
Ecuador/Loja and Zamora-Chinchipe	Stems, leaves	Infusion	Relaxant, insomnia	[42]
Ecuador/Loja	Whole plants, branches	Crushed	Nerves	[43]
Greece/Macedonia	Leaves of *Melissa* officinalis subsp. altissima (Sm.) Arcang.	Decoction or infusion	As sedative; used as a decoction in combination with Crataegus monogyna Jacq. for the prevention of cardiovascular diseases	[44]
Iraq	Leaves	Herbal tea	Diuretic, analgesic; for headache, toothache, galactogen	[45]
Iraq/Hawraman	Leaves	—	Used as a wrap in dolma preparation	[46]
Iran/Chaharmahal and Bakhtiari (Shahrekord)	Aerial parts	—	Anxiety, depression	[29]
Iran/North Khorasan	Flowers, leaves	Infusion	To strengthen the memory, nerve tonic, hypnotic, antistress, sedative, anticonvulsive	[47]
Iran/Fars (Arjan-Parishan)	Leaves, seeds	Decoction	Sedative	[48]
Iran/Sistan, Baluchistan	Leaves	Decoction	Diuretic, sedative	[49]
Iran/Kermanshah	Aerial parts	Decoction	Antihistamine and antipruritus, diabetes control	[50]
Italy/Campania (Benevento Sannio)	Leaves, flowers	—	Antispasmodic, antihysteric, and tonic	[51]
Italy/Umbria	Leaves, shoots	—	Alcoholic beverages; boiled; fried in fat, without or with beaten eggs, risotto	[33]
Italy/marches	Leaves	Compress of crushed fresh leaves	To heal insect bite	[52]
Italy/Valvestino	Leaves	Poultice	Wound healing	[53]
Italy/Abruzzo, Lazio, Molise National Park	Aerial parts, leaves	Decoction	The decoction is used to favour digestion, lower blood pressure and for calming (also in case of emotional illness)	[54]
		—	An aromatic herb used as a beef condiment	
Italy/Sardinia	Leaves	Tea	Helps relieve premenstrual symptoms	[55]
	Herb	—	Nervous agitation, sleeping problems, functional gastrointestinal complaints, menstrual cramps, and urinary spasms	
Italy/Salento	Leaves	—	Seasoning in many dishes	[56]
Jordan	Aerial parts	Infusion	Sedative, carminative, antispasmodic, and digestive	[57]
Jordan	Aerial parts	—	Abdominal pain, gynaecological disorders, arthritis	[58]
Kosovo/Pejë and Deçan	Areal parts	Infusion	For treating abdominal pains during pregnancy	[59]
		Decoction	Neuro-relaxant	
	Leaves	—	Strengthen the heart, migraine, stomach disorders and memory	[60]
Lebanon/Jabal Moussa Bioreserve	—	—	Harvested as a spice, herbal tea, condiment, medicinal plant and perfumes	[32]
Macedonia	Aerial parts (fresh)	Decoction	Nervous system, focus, concentration, and relaxation, used as a spice	[61]
Morocco/Ksar Lakbir	Aerial parts	Infusion	As spasmolytic, depurative and cholagogue	[62]
Morocco/	Whole plants	—	Anti-diarrhea, astringent, febrifuge	[63]
Peru/Ancash	Leaves	Infusion	Sedative and hypotensive	[25]
Portugal/Trás-os-Montes	Aerial parts, stems, flowers, fresh or dried.	Infusion	Relaxation (nervousness, insomnia, spasms and nervous indigestion); intestinal gases and pain; digestion and bile stimulation; fever, headache and influenza; stomach ache and gastritis; for the heart; memory stimulation.	[64]
Republic of Macedonia/Sharr Mountain	Leaves	Tea, essential oil	Heart problems, headaches	[65]
Russia	Herb	Infusion	To stimulate the appetite and gastrointestinal tract; for nausea, vomiting, painful menstruation, cardiac neurosis	[66]
Serbia/Kopaonik Mountain	Aerial parts	Tea	Sedative, relaxing, digestive properties; internally taken for nervous anxiety, depression, tension headaches and indigestion (tea taken after meal)	[67]
Spain/Alava (Valdegovía, Valle de Arana, Izki)	Aerial parts	Infusion	Bronchitis, stomach pain	[68]
		Herbal tea: aerial parts, infusion, alone or with Hypericum perforatum	Relaxant, depression	
		Decoction	Stomach diseases, nephritis, cardiovascular diseases, forgetfulness, diabetes, cold, flu, bronchitis, enteritis	
Turkey/K. Maras	Leaves	—	Antiseptic, cold, diabetes, antispasmodic	[69]
Turkey/Bayramic	Leaves	Infusion	Heart diseases	[70]
Turkey/Antakya	Aerial parts *Melissa officinalis* L. subsp. *inodora* Bornm.	Decoction	Stomach pains, gastritis, ulcer, sedative	[71]
Turkey/Kumluca (Antalya)	Aerial parts of *Melissa officinalis* L. subsp. *officinalis*	Infusion	Relaxing, stomach disorders, intestinal disorders, cardiovascular disease, digestive, diarrhea, migraine, analgesic	[72]
Turkey/Anatolia	Leaves of *Melissa officinalis* subsp. *officinalis*	Decoction as tea and oils are applied to the pain region	Sedative	[73]
Turkey/Uzunköprü	Aerial parts	Infusion	Diabetes, cold, insomnia	[74]
Turkey/Samsun (Yeşilırmak Delta)	Leaves of *Melissa officinalis* subsp. *officinalis*	—	Soothes insect bite, headache, indigestion, nausea, sedative	[75]
Turkey/Osmaniye (Bahçe and Hasanbeyli)	Aerial parts of *Melissa officinalis* L. subsp. *inodora* Bornm	Infusion	Sedative, gastric and carminative	[76]
Turkey/Kahramanmaras (Andirin)	Aerial parts of *Melissa officinalis* L. subsp. *inodora* Bornm	Infusion, decoction	Pain in head, cardiac, stomach and intestinal disease	[77]
Uzbekistan/Tashkent (Chatkal Biosphere Reserve)	Whole plants	—	Epilepsy, mental illness, diuretic, digestive, fevers and colds, indigestion associated with nervous tension, hyperthyroidism, depression, mild insomnia, epilepsy, headaches, toothaches, flatulence, colic, nausea, nervousness, anaemia, vertigo, syncope, malaise, asthma, bronchitis, amenorrhea, cardiac failure, arrhythmias, depression, psychosis, hysteria, ulcers, wounds, against Alzheimer disease, sedative, anti-inflammatory, hepatoprotective, digestive, antiviral, antilipidaemic, anxiolytic	[78]

The article "Phytochemical Constituents, Biological Activities, and Health-Promoting Effects of the Melissa officinalis" was retracted in 2024. Reasons: signs of a paper mill; compromised peer review; unreliable results or conclusions.

**Table 2:** Clinical studies of *Melissa officinalis*.

Design	Observations	Country	Ref
Randomized, double-blind, placebo-controlled	In this study, the effect of *M. officinalis* supplementation was evaluated on borderline hyperlipidemia patients. The herbal capsule of *M. officinalis* extract showed significant results in hyperlipidemic patients. It reduced the level of low-density lipoprotein (LDL) and aspartate transaminase (AST) at the dose of 500 mg (two capsules of *M. officinalis* three times per day up to 2 months) (trial registration number: IRCT2014042017347N1).	Iran	[138]
Randomized, crossover trial, placebo-controlled	In this study, investigations on safety, tolerability, and pharmacokinetics of a single dose of *M. officinalis* extract were performed. A single dose of *M. officinalis* extract containing 500 mg rosmarinic acid seems to be safe and tolerable in healthy individuals. It does not affect liver, kidney, and blood cell functions, and no harmful effects were reported during this study by the patients (trial registration number: UMIN000004997).	Japan	[139]
Randomized, double-blind, placebo-controlled	In this study, the effect of *M. officinalis* extract was assessed against heart palpitation. Leaf extract of *M. officinalis* (500 mg two times per day up to 14 days) significantly reduced the incidence of palpitation and the number of anxious patients. It showed safe and beneficial effects in the treatment of palpitation patients, and no side effects were recorded during this study (trial registration number: IRCT2013012712303N1).	Iran	[111]
Prospective pilot study, single-center, open-label	In this study, the effects of Cyracos (standardized extract of *M. officinalis)* were evaluated against anxiety disorders and sleep disturbance. Chronic administration of leaf extract of *M. officinalis* (600 mg per day up to 15 days) reduced the stress-related effects including anxiety manifestations (18%), ameliorated anxiety-associated symptoms (15%), and insomnia (42%).	France	[140]
Randomized, double-blind, placebo-controlled	In this study, the effect of *M. officinalis* oil was estimated against agitation in Alzheimer's disease. Aromatherapy with *Melissa* oil was not effective compared to the known drug (trial registration number: EudraCT23148/0001/001-0001).	UK	[141]
Randomized, double-blind, placebo-controlled	In this study, anxiolytic effects of the herbal combination were evaluated during the laboratory-induced stress. *M. officinalis* (80 mg) and *Valeriana officinalis* (120 mg) were used as a combination, and their 600 mg dose improved the negative effects of the defined intensity stressor simulation on ratings of anxiety.	UK	[142]
Randomized, double-blind, placebo-controlled	In this study, the effectiveness and side effects of *M. officinalis* with two other herbs were evaluated against infantile colic. After the 1-week treatment of the herbs, crying time was reduced in 85.4% of subjects compared to control (48.9%) and no side effects were recorded during the study.	Italy	[143]
Randomized, double-blind, placebo-controlled	In this study, the effects of *M. officinalis* on laboratory-induced psychological stress were investigated. The 600 mg dose of herbal extract reduced the negative mood effects of the defined intensity stressor simulation and increased the self-ratings of calmness.	UK	[144]
Randomized, double-blind, placebo-controlled	In this study, the effects of *M. officinalis* on modulation of mood and cognitive performance were evaluated. The results indicated that doses of *Melissa* at or above can improve cognitive performance and the dose of 1600 mg showed the best results.	UK	[145]
Randomized, double-blind, placebo-controlled	In this study, the efficacy and safety of *M. officinalis* extract were evaluated in mild to moderate Alzheimer's disease patients. After the 4-month treatment, herbal extract (60 drops per day) showed a significant outcome on cognitive function compared to control.	Iran	[113]
Randomized, double-blind, placebo-controlled	In this study, the effects of *M. officinalis* were investigated against herpes simplex infections and the results suggested that the ingredient of the *Melissa* gave protection against herpes simplex infections and early-stage treatment revealed itself as most effective.	Germany	[146]

The article "Phytochemical Constituents, Biological Activities, and Health-Promoting Effects of the Melissa officinalis" was retracted in 2024. Reasons: signs of a paper mill; compromised peer review; unreliable results or conclusions.

## Data Availability

The data supporting this review are from previously reported studies and datasets, which have been cited. The processed data are available from the corresponding author upon request.
